This article has been retracted.

# Adoption of Compound Echocardiography under Artificial Intelligence Algorithm in Fetal Congenial Heart Disease Screening during Gestation

**DOI:** 10.1155/2022/6410103

**Published:** 2022-06-01

**Authors:** Guowei Han, Tianliang Jin, Li Zhang, Chen Guo, Hua Gui, Risu Na, Xuesong Wang, Haihua Bai

**Affiliations:** ^1^Department of Ultrasonography, Affiliated Hospital of Inner Mongolia Minzu University, Tongliao, 028000 Inner Mongolia, China; ^2^Inner Mongolia Engineering and Technical Research Center for Personalized Medicine, Tongliao, 028000 Inner Mongolia, China; ^3^Department of Obstetrics, Affiliated Hospital of Inner Mongolia Minzu University, Tongliao, 028000 Inner Mongolia, China; ^4^Genetic Testing Center, Affiliated Hospital of Inner Mongolia Minzu University, Tongliao, 028000 Inner Mongolia, China; ^5^College of Life Sciences and Food Engineering of Inner Mongolia Minzu University, Tongliao, 028000 Inner Mongolia, China

## Abstract

This research was aimed at exploring the diagnostic and screening effect of composite echocardiography based on the artificial intelligence (AI) segmentation algorithm on fetal congenital heart disease (CHD) during pregnancy, so as to reduce the birth rate of newborns with CHD. A total of 204 fetuses with abnormal heart conditions were divided into group II, group C (optimized with the AI algorithm), and group W (not optimized with the AI algorithm). In addition, 9,453 fetuses with normal heart conditions were included in group I. The abnormal distribution of fetal heart and the difference of cardiac *Z* score between group II and group I were analyzed, and the diagnostic value of group C and group W for CHD was compared. The results showed that the segmentation details of the proposed algorithm were better than those of the convolutional neural network (CNN), and the Dice coefficient, precision, and recall values were higher than those of the CNN. In fetal CHD, the incidence of abnormal ultrasonic manifestations was ventricular septal defect (98/48.04%), abnormal right subclavian artery (29/14.22%), and persistent left superior vena cava (25/12.25%). The diagnostic sensitivity (75.0% vs. 51.5%), specificity (99.6% vs. 99.2%), accuracy (99.0% vs. 98.2%), negative predictive value (88.5% vs. 78.5%), and positive predictive value (99% vs. 57.7%) of echocardiography segmentation in group C were significantly higher than those in group W. To sum up, echocardiography segmented by the AI algorithm could obviously improve the diagnostic efficiency of fetal CHD during gestation. Cardiac ultrasound parameters of children with CHD changed greatly.

## 1. Introduction

Congenital heart disease (CHD) is a birth defect that causes structural and functional abnormalities of the heart and blood vessels at birth, which is the most ubiquitous congenital disease that affects the health of infants [1]. According to the statistics of the World Health Organization (WHO), about 1.49 to 2.01 million infants are born with CHD every year [2]. CHD accounted for 1.2% of newborns in the United States [3]. However, the incidence of neonatal CHD in China is 1.36%, with significant regional differences [4]. CHD belongs to the normal range of congenital malformation, and the occurrence factors are directly related to chromosome abnormality. CHD is a major cause of death in newborns and children. With the growth of fetus, the heart and blood vessels develop in disorder. Hence, the fetuses' heart and blood vessels have various levels of problems in many ways, and there are even severe stillbirth and miscarriage. Although surgical treatment can alleviate the disease in children with CHD, survival is relatively short. Therefore, early diagnosis of CHD during gestation is of great significance [5].

Echocardiography has long become the first choice for the diagnosis of CHD because it is noninvasive, nonradiative, real-time imaging, and low-cost. In the echocardiography, the two most pervasively used scans are apical four-chamber view and apical two-chamber view. From these two parts, the sonographer examines structures of the ventricles and atria [6]. By dividing the left ventricle on these two sections, the physician measures some vital clinical indexes, such as left ventricular end-systolic volume (LVESV) and left ventricular end-diastolic volume (LVEDV). Then, the ejection fraction is calculated, which is the major index to evaluate the cardiac function. Besides, it is very important for the diagnosis of CHD. Nevertheless, manual segmentation of the left ventricle is extremely dependent on the physician's expertise and clinical experience, which is a waste of time and energy and greatly increases the workload of the physician [7]. Therefore, the computer-aided diagnosis technology is applied, and crucial anatomical structures are automatically segmented, thus further freeing physicians from heavy and repetitive work.

Medical image segmentation is a vital topic in medial image procession and analysis, as well as the considerable steps of subsequent medial image analysis. Traditional medical image segmentation is mainly controlled by physicians' experience. With the pervasiveness of computer-aided diagnosis, it is applied to medical image segmentation gradually. In recent years, machine learning methods, especially deep learning methods based on convolutional neural networks (CNNs), have made remarkable breakthroughs and achievements in the field of computer vision. These methods are also applied to medical image segmentation [8]. With the emergence of U-Net network, the research and adoption of the deep learning method under the deep CNN in medial image segmentation have attracted much attention [9]. Based on the analysis of the content of echocardiography, the adoption of deep CNN in medical segmentation was discussed. The adoption of the technology in the screening of fetal congenital heart disease was investigated during gestation under the compound echocardiography based on the AI segmentation algorithm. Additionally, a new method for fetal CHD screening during gestation was provided.

This study was aimed at exploring the value of composite echocardiography in screening for maternal and fetal CHD and to improve the quality of life of newborns. The pregnant women were selected as research subjects, and fetal composite echocardiograms were collected. In addition, artificial intelligence (AI) segmentation algorithms were adopted to segment the regions of interest (ROI) in the composite echocardiograms and the value of segmented images for screening fetal congenital heart disease (CHD) during pregnancy. This study was intended to provide the possibility to improve the accuracy of early screening of fetal coronary heart disease in clinic.

## 2. Materials and Methods

### 2.1. Research Object

The pregnant women who underwent fetal ultrasound cardiac screening in combination with other procedures at the hospital between January 2017 and December 2021 were included in this research. 204 fetuses with cardiac abnormalities by ultrasound screening combined with other examination methods were set as group II. According to the result standard, the composite ultrasound images were divided into group C (optimized by the AI algorithm) and group W (not optimized), including 204 cases. Then, 9,453 fetuses with normal heart disease in hospital were selected as group I. The abnormal distribution of the fetal heart and the difference of cardiac *Z* score between group II and group I were analyzed, and the diagnostic value of group C and group W for CHD was compared. The study had been approved by the ethics committee of hospital, and families of the whole patients signed the informed consent.

### 2.2. Color Doppler Ultrasound Scan

Color Doppler ultrasonography was employed for examination. A routine obstetric ultrasound was performed firstly. Then, the fetal heart structure was tested. The content of general obstetric ultrasound examination was determining the number of fetuses. The fetal head circumference, diameter of double parietal bone, and fetal heart structure were mainly observed and measured from the fetal heart. Four-chamber view, long axis of right ventricle, and pulmonary artery were observed and measured. During the examination, if the section was not clear, the puerpera needed to be examined again after the proper exercise. Besides, if the effect was not ideal, it should choose another day to do the examination until the section was clear.

### 2.3. AI Algorithm Segmentation Image

The major task is exactly segmenting the left ventricle and left atrium in the image of the four-chamber apical view and the two-chamber apical view. The examples of deep CNNs and convolutional block attention modules for natural image segmentation were considered. Then, a compound echocardiography segmentation network under the AI algorithm was proposed to segment echocardiography. In Figure 1, echocardiography was composed of spatial branch network and context branch network and feature fusion module. Moreover, convolutional block attention module was added into each network branch, which consisted of space attention submodule and channel attention submodule. The spatial attention submodule helped guide the learning of network feature by learning the spatial relations of features. The characteristic graph *T*_*c*_ output by the intermediate layer was given. Firstly, maximum pooling and average pooling were performed by channel direction. Two pooled results were pieced together based on channels. Then, the spatial features of the input feature graph were aggregated. After the aggregation features were input into the convolutional layer, the attention force diagram *N*_*c*_ in two-dimensional space was obtained. Finally, the extracted feature *T*_*c*_′ was obtained by the dot product of the input characteristic *T*_*c*_ and the spatial attention force *N*_*c*_, that was, the equation (1).

(1) $$\begin{array}{c} T_{c}^{\prime }=T_{c}*N_{c}. \end{array}$$

Therefore, the spatial attention submodule could mine the spatial relations in the feature graph and further focus on where there was the noteworthy features and information. The number of neurons in the hidden layer to *D/i* was set to reduce the number of parameters, where *D* represented the number of input feature graphs and *i* represented the attention coefficient. After multilayer perceptron was processed, it was obtained that the two eigenvectors were added element by element for fusion. Then, the weighted eigenvector *N*_*d*_ was obtained by softmax operation. Eventually, the extracted feature *T*_*d*_′ was obtained by multiplying the input feature *T*_*d*_ and the eigenvector *N*_*d*_ in equation (2).

(2) $$\begin{array}{c} T_{d}^{\prime }=T_{d}*N_{d}. \end{array}$$

The normal crossentropy loss function was used to train the proposed AIDAN network. An auxiliary loss function was added to supervise the training of context branch networks. Under the main loss function, two auxiliary loss functions were employed to supervise the training of the context branch network in the last two downsampling stages. Specifically, the adopted loss function was equation (3).

(3) $$\begin{array}{c} A\left(V;U\right)=A_{q}\left(V;U\right)+b_{1}A_{1}\left(V_{1};U\right)+b_{2}A_{2}\left(V_{2};U\right). \end{array}$$

In equation (3), *A*_*q*_ represented the primary loss function, and *V* represented the prediction of the final output of the entire network. *U* represented the learnable parameter of the network, and *A*_1_ and *A*_2_ represented the auxiliary loss functions of the final two down-sampling stages of the context branch network, respectively. *V*_1_ and *V*_2_ represented the feature graphs output in the last two downsampling stages of the context branch network. The weights before the main loss function and the two auxiliary loss functions were determined by *b*_1_ and *b*_2_. There was the equation (4).

(4) $$\begin{array}{c} b_{1}=b_{2}=1. \end{array}$$

The use of joint loss function helped the model to be better optimized and trained.

### 2.4. Evaluation Indexes of Segmentation Effect

Dice coefficient, precision, and recall were calculated to evaluate the segmentation effect.

Dice coefficient was used to evaluate the difference of the overlap between the segmentation results and the annotation results from experts. The larger the Dice coefficient was, the better the segmentation effect was. Equation (5) was the Dice coefficient calculation equation.

(5) $$\begin{array}{c} \text{Dice}=\frac{2\times \text{Correct prediction}}{\text{True results}+\text{Prediction resluts}}. \end{array}$$

Precision ratio was used to evaluate the proportion of the correct classification results. The higher the precision value was, the better the closer the segmentation result was to the truth. Equation (6) was the equation for precision ratio.

(6) $$\begin{array}{c} \text{Precision}=\frac{\text{True prediction}}{\text{True prediction}+\text{False prediction}}. \end{array}$$

Furthermore, recall ratio was used to evaluate the proportion of the correctly classified pixels to total pixels. The larger the recall value was, the closer the segmentation result of the algorithm was to the truth. Equation (7) was the calculation of recall ratio.

(7) $$\begin{array}{c} \text{Recall}=\frac{\text{True prediction}}{\text{True prediction}+\text{False negative}}. \end{array}$$

### 2.5. Methods for Evaluation of Diagnostic Effectiveness

Diagnostic sensitivity, specificity, accuracy, negative predictive value, and positive predictive value were used to calculate the diagnostic results of the two groups of examination methods, and the specific calculation methods were shown in Table 1.

### 2.6. Statistical Analysis

SPSS 18.0 was employed to compare the results of pregnant women examinations between the two groups. Frequency (%) was used to show the enumeration data, and *χ*^2^ test was used to compare the difference. Measurement data were presented by using *mean* ± *standard* *deviation*, and differences were compared by using the independent sample *t*-test. The difference was statistically significant in the index data between the two groups with *P* < 0.05.

## 3. Results

### 3.1. Comparison of Basic Data between Two Groups of Pregnant Women

The differences between the two groups of basic data of pregnant women were collected and compared (Table 2). There was no significant difference between group I and group II in such aspects as average age, average gestation, and average number of births (*P* > 0.05).

### 3.2. Evaluation of Segmentation Effect of Compound Echocardiography

The effect of the proposed algorithm on the segmentation of fetal echocardiography with abnormal cardiac structure was evaluated (Figure 2). Compared with the traditional CNN algorithm, the proposed algorithm had better segmentation effect of abnormal structure, and it could better identify and segment the details.

The Dice coefficient, precision, and recall were used to quantitatively evaluate segmentation effect of cardiac abnormal structures through CNN algorithm and the proposed algorithm. In Figure 3, the Dice coefficient (0.93), precision (0.95), and recall (0.92) of the AI algorithm were totally higher than those of the CNN algorithm (0.91, 0.92, and 0.90, respectively).

### 3.3. The Type Distribution of Fetal CHD

Figure 4 shows the distribution of disease types in 204 fetuses with cardiac abnormalities. There were 25 fetuses (12.25%) with persistent left superior vena cava, 98 (48.04%) fetuses with ventricular septal defect, 6 fetuses (2.94%) with single ventricle, and 3 fetuses (1.47%) with single atrium. The 29 fetuses (14.22%) had abnormal right subclavian artery. 3 fetuses (1.47%) had transposition of the great arteries, and 2 fetuses (0.98%) had interrupted aortic arch. There were 6 fetuses (2.94%) with aortic coarctation, 8 fetuses (3.92%) with right-sided arcus aorta, 1 fetus (0.49%) with absence of inferior vena cava, 11 fetuses (5.39%) with pulmonary artery stenosis, 5 fetuses (2.45%) with endocardium pad defect, 1 fetus (0.49%) with persistent truncus arteriosus, 1 fetus (0.49%) with pulmonary artery atresia, and 5 fetuses (2.45%) with double-outlet right ventricle. The proportion of ventricular septal defect, persistent left superior vena cava, and abnormal right subclavian artery is relatively high, followed by pulmonary artery stenosis and right anus (Figure 5).

### 3.4. Value Analysis of Echocardiography in Fetal CHD before and after Segmentation

Figure 6 shows the sensitivity, specificity, accuracy, negative predictive value, and positive predictive value of echocardiography in the diagnosis of fetal CHD in group C and group W. It illustrated that the diagnostic sensitivity (75.0% vs. 51.5%), specificity (99.6% vs. 99.2%), accuracy (99.0% vs. 98.2%), negative predictive value (88.5% vs. 78.5%), and positive predictive value (99% vs. 57.7%) of echocardiography segmentation in group C were significantly higher than those in group W.

## 4. Discussion

There are approximately 115,000-199,000 newborns in China who suffer from CHD every year. The survival rate of these newborns is low, and the neonatal mortality rate is high. Fetuses with CHD present small head circumference, normal posterior fossa measurements, and low birth weight [10]. More so, pregnant patients with fetuses affected by CHD present increased risk of abnormal pregnancy outcomes in terms of preterm delivery and preeclampsia, particularly [11]. Fetal movement and gestational age are closely related to the accuracy of ultrasound examination for the fetal heart. Therefore, choosing the right time for inspection is of great significance [12]. Color Doppler ultrasound is the most ideal way to examine fetal cardiac structure. During the second trimester of pregnancy, cardiovascular problems are often detected. Hence, in China, fetal congenital diseases are usually screened during the second trimester of pregnancy [13]. After the fetal congenital diseases are screened, detailed examination and treatment methods need to be further developed [14]. Early screening is of great significance because screening fetal CHD in the middle of pregnancy is not conductive to later diagnosis and treatment. At present, screening fetal heart disease is generally performed at 18-22 weeks of gestation, and the effect is relatively ideal [15]. It is difficult for small fetal heart to examine the echocardiography at 19 weeks; so, the rate of misdiagnosis or missed diagnosis is high. Furthermore, the development of the fetal heart is relatively complete at 19-26 weeks of gestation. When the fetal heart develops to a certain extent, fetal activity is more active, and different parts and structures of the heart can be visualized clearly. Hence, processing is much easier at this stage [16]. Based on this, it was hoped to improve the diagnostic value of echocardiography in fetal CHD.

About 91% of congenital heart disease is influenced by environmental factors and genetic factors. The risk factors of fetal congenital heart disease screening by ultrasound usually come from the fetus itself, pregnant women, and genetics, including medically assistance reproduction. The risk factors of fetal CHD include puerpera (gestational hypertension, teratogenic drugs, and immune diseases), fetus (chromosomal abnormalities and edema), and family history (CHD and birth malformations) [17, 18]. 9,657 pregnant women were included, of which 204 fetuses had heart abnormalities, with a detection rate of 2.1%. Echocardiography is the main clinical method for screening fetal CHD due to the high safety because it can clearly show the ventricle and atrioventricular value [19, 20]. In fetal CHD, the largest proportion was ventricular septal defect (98/48.04%), followed by aberrant right subclavian artery (29/14.22%), and the last was persistent left superior vena cava (25/12.25%). The aberrant right subclavian artery is the failure of the right subclavian artery and the left common carotid artery to confluence due to various factors during the fetal period, leaving the right subclavian artery and causing vascular malformation. This change is a benign change, but it cannot be recovered by itself [21]. Therefore, echocardiography was used to evaluate and identify fetal heart abnormalities [22]. Subsequently, the adoption of echocardiography technique in screening fetal CHD during gestation was investigated under the compound echocardiography based on the AI segmentation algorithm. After segmentation, the Artificial intelligence algorithm sends a large number of scans for reevaluation and needs to handle additional workload, but the results showed that the diagnostic sensitivity (75.0% vs. 51.5%), specificity (99.6% vs. 99.2%), and accuracy (99.0% vs. 98.2%) of the echocardiogram after segmentation were markedly higher than those before segmentation. The above research results confirmed that the AI algorithm proposed in this work showed obviously predictive value in fetal CHD after the segmentation of the composite echocardiogram [23]. The results showed that the AI algorithm can improve the accuracy of ultrasonic image in disease diagnosis and has good application value. Sun et al. (2021) [24] concluded that the bilateral filtering intelligent denoising algorithm can improve the diagnostic value of ultrasound elastography for cervical intraepithelial neoplasia (CIN). Luo et al. (2021) [25] also reached a consistent conclusion and gave certain support to this study. Furthermore, the good development prospect of the AI algorithm in medical image processing is proposed.

## 5. Conclusion

It investigated the diagnostic and screening effects of composite echocardiography based on the AI segmentation algorithm for fetal CHD during pregnancy in this work. The results showed that AI algorithm segmentation echocardiography could significantly improve the diagnostic efficiency of fetal CHD during pregnancy, and there were significant changes in cardiac ultrasound parameters of children with CHD, which was convenient for clinical screening. However, the sample size of this study is small, and it should include more people in the experiment. Moreover, clinical trials are not implemented in a single area or in a small area but in multicenter and large-sample hospitals. However, through research, it can fully understand that the AI algorithm in medical image processing had a good development prospect, worthy of further clinical exploration.

## Figures and Tables

**Figure 1:** Double network echocardiography segmentation model.

**Figure 2:** Segmentation of abnormal cardiac structures. (a) showed the original echocardiogram, (b) showed the segmentation effect of the CNN algorithm, and (c) showed the segmentation effect of the AI algorithm (the red curvilinear area referred to the segmented location of the lesion).

**Figure 3:** Quantitative indexes of segmentation effect of cardiac abnormal structure.

**Figure 4:** The disease type distribution of CHD in fetuses. (a) Persistent left superior vena cava. (b) Ventricular septal defect. (c) Single ventricle. (d) Single atrium. (e) Abnormal right subclavian artery. (f) Transposition of the great arteries. (g) Interrupted aortic arch. (h) Aortic coarctation. (i) Right-sided arcus aortae. (j) Absence of inferior vena cava. (k) Pulmonary artery stenosis. (l) Endocardium pad defect. (m) Persistent truncus arteriosus. (n) Pulmonary artery atresia. (o) Double-outlet right ventricle.

**Figure 5:** Ultrasonic images of fetus with abnormal heart. (a) Persistent left superior vena cava. (b) Ventricular septal defect. (c) Abnormal right subclavian artery. (d) Pulmonary artery stenosis. (e) dextroaortic arch.

**Figure 6:** Diagnostic value of echocardiography before and after segmentation.

**Table 1:** Calculation method of diagnostic effect evaluation indicators.

Indicator	Calculation method
Sensitivity	*Sample* *number* *consistent* *with* *actual* *positive* *results*/*total* *sample* *number* × 100%
Specificity	*Number* of *samples* *consistent* *with* *actual* *negative* *results*/*total* *number* of *samples* × 100%
Accuracy	(*number* of *samples* *with* *positive* *results* + *number* of *samples* *with* *negative* *results*)/*total* *sample* *number* × 100%
Negative predictive value	*Number* of *samples* *consistent* *with* *actual* *negative* *results*/*total* *number* of *samples* *tested* *negative* × 100%
Positive predictive value	*Number* of *samples* *consistent* *with* *actual* *positive* *results*/*total* *number* of *samples* *tested* *positive* × 100%

**Table 2:** Comparison of basic data between the two groups of pregnant women.

Group	Age (years old)	Gestational age (weeks)	Number of births (times)
Group I (*n* = 9,453)	28.03 ± 2.15	12.35 ± 0.55	1.08 ± 0.22
Group II (*n* = 204)	27.79 ± 3.04	12.18 ± 0.41	1.12 ± 0.30
*t*	-0.155	0.121	-0.037
*P*	0.978	0.744	0.826

## Data Availability

The data used to support the findings of this study are available from the corresponding author upon request.
